# Exploring the convergence of ICT, digital financial inclusion, environmental pressures, and free trade and their significance in driving sustainable green investment initiatives under carbon neutrality targets

**DOI:** 10.1016/j.heliyon.2024.e31102

**Published:** 2024-05-10

**Authors:** Jianmin Zhu, Wei Yan, Junliang He, Muhammad Hafeez, Sidra Sohail

**Affiliations:** a Institute of Logistics Science and Engineering, Shanghai Maritime University, Shanghai, China; b China Institute of FTZ Supply Chain, Shanghai Maritime University, Shanghai, China; c Adnan Kassar School of Business, Lebanese American University, Beirut, Lebanon; d Pakistan Institute of Development Economics (PIDE), Islamabad, Pakistan; e Institute of Business Management Sciences, University of Agriculture, Faisalabad, Punjab, Pakistan

**Keywords:** ICT, Digital financial inclusion, Environment pressure, Free trade, Green investment, Carbon neutrality targets

## Abstract

Due to its rapid economic development over the past few decades, China is now at the forefront of environmental issues, necessitating creative solutions that combine ICT, digital financial inclusion, environmental pressure, and free trade to encourage green investment. This study aims to investigate the linkage between ICT, digital financial inclusion, environmental pressure, free trade, and green investment in China from 1996 to 2022 by employing the Partial least squares structural equation modelling (PLS-SEM). As per our results, the statistical values of Cronbach's alpha, composite reliability, and average variance are all above the cutoff point, demonstrating the applicability of this methodology. According to the structural model's results, the path coefficients between digital financial inclusion and green investment, environmental pressure and green investment, and GDP and green investment are positively significant, implying that these three factors are crucial for boosting green investment in China. In addition, our vector autoregressive model results suggest that ICT, digital financial inclusion, environmental pressures, free trade, and GDP cause green investment to rise in China. Thus, the policymakers in China should focus on developing comprehensive policies to encourage green investment in China, which is crucial for economic and environmental sustainability.

## 1 Introduction

The main strategy for addressing the issue of worldwide contamination of the environment is to enhance green investment. Economic globalization has been the primary engine for the world's economic expansion and social advancement in recent years due to its consistent promotion of the rise of international trade and foreign investment. Environmental contamination is widespread, nevertheless, and resource shortages and environmental issues have grown more apparent with fast economic expansion [1,2]. China has the worst environmental contamination of all the emerging nations. The economy of China has been expanding at a pace of around 10 % for many years. Nevertheless, its rapid economic growth has resulted in instances of environmental damage [3]. Coordinating the interaction between the economy and the environment is a current social problem. Investment in green technologies concentrates on synergistic growth; it seeks to increase the effectiveness of resource consumption and decrease pollutants released in the entire manufacturing process, contributing significantly to the integrated advancement of the economy and sustainability [4]. Nevertheless, the intricate and distinctive nature of green investment, as well as the immaturity of the green market, result in higher costs, increased market risks, and longer investment return cycles [5], leading to significant financial constraints in the enhancement of green investment.

Innovative finance models may aid in removing the barriers preventing rapid green investment. These financial frameworks must deal with the old banking industry's improper allocation of financial resources [6]. The fast progress of digital technology offers fresh suggestions for supply-side reform, which coincides with the fast growth of financial technology [7]. The door has been opened for the digitalization of inclusive finance due to the Internet's quick growth in the financial industry. In today's world, inclusive finance is a key idea for putting the emerging idea of development into reality, for creating an innovative development arrangement, and as a powerful tool for advancing social fairness and achieving shared prosperity [8]. Without altering the fundamental financial responsibilities of payment clearing, capital funding, and risk mitigation, it primarily concerns technological advancements in transaction pathways, transaction procedures, and transaction platforms. The major difference between digital and conventional finance depends on the channels through which both modes work. Digital finance relies on digital channels, including big data, cloud computing, blockchain, and artificial intelligence [9]. As the end result of the thorough fusion of the new technology revolution with financial reform, inclusive digital finance may support the growth of green finance and foster corporate green innovation by lowering the cost of financial services, encouraging the restructuring of the consumption structure and enhancing the effectiveness of capital allocation. Green investment continues to be in the exploratory phase as an essential goal to safeguard the environment and encourage sustainable economic and societal growth [10]. The growth of green investment may be sped up and made more effective with the help of digital inclusive finance. On the one hand, via technological transfer, digital finance may assist green financial organizations in lowering transaction costs and the potential for default and increasing the effectiveness and return of green lending [11]. On the other hand, it may expand the green financial sector via platform integration, provide a wider variety of green financial goods, and create a win-win scenario where the financial sector is greatly enhanced and sustainable economic growth is achieved [12].

The internet revolution is the primary reason behind the digitalized and more inclusive financial system. ICT directly impacts green investment in this age of digitalization. By lowering social, technical, and informational barriers, the ICT sector assists governments in advancing clean energy sources and ecologically beneficial energy initiatives [13]. People's behaviour has changed due to the growth of ICT, moving from offline to online, which may open up new opportunities for adopting sustainable energy. On the one hand, increased social network accessibility will increase public awareness of environmental preservation efforts and promote information and technology exchange between businesses in the United States and overseas. It increases public awareness of and enthusiasm for green technology and sustainable energy sources [14]. ICT, on the other hand, is crucial for facilitating and accelerating green investment since it offers the necessary tools, platforms, and procedures. ICT also facilitates data collection, analysis, and distribution, giving investors important knowledge about carbon footprints, use trends, and evaluations of environmental consequences. With this information, investors may make well-informed choices, spot possible green investment possibilities, and evaluate environmental and economic dangers [15]. Further, ICT platforms and online markets also link financiers to green initiatives, enhancing market availability and transparency [16]. These networks allow investors to research various renewable energy ideas, assess their financial potential, and contribute to green projects.

In addition to financial development and ICT, some other factors, such as trade liberalization and environmental degradation, may also impact green investment [17]. Free trade agreements make it easier to reach worldwide markets, which motivates companies to look for commercial possibilities abroad for green goods and technology. Investments in green industries, including clean technology, sustainable agriculture, and renewable energy, might benefit from this increased market access [18]. Innovation in green technology may be fueled by competition, which is encouraged by free trade. Moreover, companies often spend money on research and development to produce environmentally friendly goods and procedures to stay competitive in the global market [19]. On the other side, businesses are compelled to invest in green technology and practices by stricter environmental rules and standards, which are often implemented in reaction to growing environmental challenges. Failure to comply may result in legal problems, penalties, and reputational harm [20].

Carbon neutrality goals are set by the world community as the best possible option to achieve superior environmental quality. The world community has pledged to achieve carbon neutrality goal by 2050; however, China stated to achieve these goals by the year 2060 [21]. China is the biggest contributor to global carbon emissions and its role is vital in achieving carbon neutrality objectives. Therefore, the policymakers in China are focusing on the factors that can help achieve carbon neutrality goals within the given timeline. Over the past few decades, the significance of green investment is well expected to reduce carbon emissions, which is vital in achieving carbon neutrality goals in China as well as globally [22]. The primary motivation of this analysis arises from comprehending the role of ICT, digital financial inclusion, environmental pressures, and free trade in fostering green investments within the framework of carbon neutrality**.**

The role of green investment is widely acknowledged as a primary contributor to clean transition and superior environmental quality in the environment-energy literature [23,24]. Despite its significance in promoting clean environment and green energy transition, it's determinants are not extensively studies in the except for the few. Since renewable energy and green innovations are used as a proxy of the green investment, most esmpirics have estimated the finance related factors as their determinants [25]. However, none of the past studies have estimated the role ICT, digital financial inlcusison, free trade, and environmental degaradtion in the green investment function of China. Therefore, this study has a research question for investigation: *What is the significance of ICT, digital financial inclusion, environmental pressures, and free trade in driving sustainable green investment?*

This study adds value to the literature in the following ways. First, as per our limited knowledge, this is the first study to examine the influence of ICT, digital financial inclusion, environmental pressure, and free trade on green investment in China. The study seeks to thoroughly explain how China's green investment landscape is formed in a dynamic and growing global environment by undertaking a holistic analysis of these numerous aspects and their linkages. Second, given China's distinct sociopolitical and economic environment, the research offers insightful details about how these elements function there. This contextual study aids in comprehending how China's unique conditions impact its strategy for green investment. Third, this study employed the Partial Least Squares Structural Equation Modeling (PLS-SEM), which helps to estimate the relationships between observed variables and latent (unobservable) constructs. Lastly, the conclusions drawn from this study may be an invaluable tool for Chinese policymakers. It offers evidence-based advice for formulating and applying regulations about sustainable development and green investments, coordinating regulatory objectives with actual results. This study has the potential to inform policy, guide business decisions, and contribute to global efforts towards environmental sustainability.

## 2 Theoretical framework

The use of ICT by businesses and firms significantly helps to foster the generation of green innovations [26], a vital component of green investment. In order to develop green innovation, it is crucial for firms to accumulate real-time data across all stages of manufacturing [27]. The implementation of information and digital technologies, specifically the incorporation of intelligent and smart devices in machinery and the complete production line, allows organizations to acquire precise information relating to each phase of production [28]. This ultimately led to enhanced production of eco-friendly innovations by fostering green investment. The link between digital financial inclusion and green innovations, investment, and revenues has come under the limelight in a growing body of contemporary studies [29]. More importantly, within the framework of green innovation, digital finance helps to enhance urban economic concentration and develop the local financial set-up. This is helpful in creating an environment that is favourable for the external financial framework, which consequently enhances green innovation in firms and enterprises by resolving their financial constraints [30]. Tang et al. [31] confirmed the positive role of digital finance in promoting green innovation within the context of new energy companies in China. Therefore, we believe that a digital and inclusive financial sector helps boost green innovations in China at the national level.

As the trade increases, the competitive environment and the opportunity to reach bigger markets may induce the firms to use greener and more sustainable technology [32]. One of the main advantages of growing trade relationships between the countries is its ability to facilitate the transfer of green technologies, knowledge, and best practices globally, enhancing an environment in which economies struggle to surpass each other in terms of sustainability [33]. Moreover, the firms increase their investment in R&D activities that promote green innovations because of accessibility to a wide variety of international markets where the demand for green innovations is high. This theoretical link sheds light on the role of trade not only in promoting economic development but also in eco-friendly innovations, which ultimately foster the demand for green investment.

Indeed, experimentation has a vital role in finding solutions to the issues of climate change and sustainability. Thus, the issues of climate change and sustainable economic development can be resolved with the help of technology transfer and innovation [34]. As the countries become more and more developed, the demand for a cleaner environment also increases, which induces policymakers to invest in green innovations and technologies. Eco-innovations are widely believed to be the most viable option to mitigate harmful environmental impacts due to large-scale economic activities [35]. Therefore, environmental deterioration increases the demand for green innovations due to their ability to mitigate the impact of climate change by laying the foundation of a low-carbon economy.

## 3 Materials and methods

Over the past several years, there has been a massive increase in the use of the “covariance-based structural equation modeling (CB-SEM)” technique which has the ability to investigate the complex linkage between recognizable and latent variables [36]. However, during this time most researchers have replaced the CB-SEM with PLS-SEM [37]. No doubt that PLS-SEM is widely recognized and employed in the field of social science. The PLS-SEM is a useful approach in the eye of empirics because it can estimate the complex models that include numerous constructs, indicator variables, and structural routes, without taking into account the distributional assumptions on the data [38]. Nonetheless, the PLS-SEM is an estimation technique that is used as a causal-predictive approach for SEM, which signifies the importance of anticipation when forming statistical frameworks whose structures are meant to offer causal linkages [39]. This method thus removes the apparent differences between description and prediction, which has become the base for generating managerial impacts and is widely recognized in the literature [40]. Moreover, to apply the PLS-SEM, some software are easy to use, e.g., PLS-Graph and Smart PLS [41], and some are more complicated and advanced, e.g., R.

While deciding between CB-SEM and PLS-SEM, we must have complete knowledge regarding the merits and demerits of both methodologies. CB-SEM is helpful when we need to validate the known theories. PLS, in contrast, is a type of predictive approach for SEM that most of the time is helpful in exploratory research. In addition, it is a good method when we are dealing with confirmatory research [42]. PLS-SEM is an efficient technique when we need to tackle the apparent division between confirmatory and predictive research. Empirics applying the approach assume that the prediction power of their model is highly accurate, alongside being strongly based on comprehensive causal explanations [43]. Below we have provided some important properties of the PLS-SEM, which makes it superior to CB-SEM.

PLS-SEM is a technique which relies on the whole variance for getting the estimates of the coefficients and is commonly known as a variance-based approach [36]. Over the last decade, the application of the PLS-SEM in different scenarios has been widely debated. Several reasons justify preferring the PLS-SEM over the CB-SEM. First, for applying CB-SEM the data must be normally distributed and big enough, while PLS-SEM has no such restrictions [44]. Second, the PLS-SEM can more clearly express the significance of the data due to its more promising statistical characteristics than CB-SEM [45]. Thirdly, the PLS-SEM has shown more strength in creating and estimating mathematical frameworks. It is an appropriate technique in authentication of causal association that has been estimated before. However, due to multicollinearity, the framework may suffer from various effects such as increasing the estimates' projected variance, making the reliability even worse. The important point is that it is quite difficult to separate the impact of special features of each independent variable on dependent variables. Thus, the problem of multicollinearity needs to be fixed. When comparing other traditional techniques such as "least squares method, principal component analysis, and ridge regression", the PLS can efficiently deal with the issue of multicollinearity [46]. In this study, we have opted for SEM strategy supplemented by the PLS; both are combined in line with the framework mentioned above.

### 3.1 Measurement model

Within this framework, we need to take the “observable variables” belong to J series, in which every set of is made of p_j_ variables. The series of “observable variables” are signified by the X_j_(X_j1_, X_j2_, …, X_jpj_) where j = 1, 2, …, J, signifies several perspectives ranging from 1-n, and every variable is intensive. These “observable variables” are not alone and are linked to a comparable latent variable, with a zero mean and variance of one standardization. To develop an outer framework or also known as a measurement model, and the standardization stated above is crucial. The outer model uses two techniques to estimate the link between the observable and latent variables. The first of the two techniques is known as “reflective technique”, in which each “observable variable X_jh_ (j = 1, 2, …, J; h = 1, 2, …, pj) is related to every single latent variable. In order to express this relationship in a linear form we develop the following model:

(1) $$X_{jh}=\lambda_{jh}\xi_{jh}+\varepsilon_{jh}$$

ε_jh_ is a white noise residual term. equation (1) is based on the following assumption:

(2) $$E\left(X_{jh}/\xi_{j}\right)=\lambda_{jh}\xi_{j}$$

This equation (2) is referred to as the “forecast-appointed” condition, based on the hypothesis revealing the zero mean residual, representing no correlation with the latent variable. There are three approaches such as “principal component analysis, Cronbach's Coefficient α, and Dillon Goldstein's rho coefficient ρ” proposed by the smart PLS3 software to investigate the reflective measurement which is a causative connection between latent and observable variables. If the observable variables don't fulfill the investigative requirements, certain variables might be removed or isolated from the group to follow the mandatory requirements. The latent variable ξj is an outcome of the linear framework of all the variables in its “observable variable” set, as shown by formative measurement.

(3) $$\xi_{j}=\sum_{h=1}^{p_{j}}WX_{jh}+\delta_{j}$$

In equation (3) we identify δj as a white noise error term. The specification (4) below is anticipated to meet the “forecast-appointed” condition:

(4) $$E\left(\xi /x_{1},x_{2},...........,x_{j}\right)=\sum_{h=1}^{p_{j}}WX_{jh}$$

In the above equation (4) δ_j_ is a white noise error term with 0 mean, implying that the error term is not linked to the observable variable X_jh_.

### 3.2 Structure model

A structural model, usually signified by the linear framework, helps define the implicit variable varied causative link is shown below**:**

(5) $$\xi_{j}=\sum_{i\neq j}\beta_{ij}\xi_{i}+\zeta_{j}$$

where the white noise disturbance term linked to “forecast appointed” condition is signified by ζj. In simple words, it means that there is no causative link between residual averages which is zero and ξj. Equation (5) reveals the presence of interdependent linkages throughout significant variables, making a causal association framework that must be a linear order of cause and effect, implying there are no circular connections within the causal framework.

### 3.3 Model estimation

In order to produce the estimated values of the latent variables, PLS utilizes iterative techniques. Firstly, it utilizes the outer estimation technique, which estimates the latent factors that rely on the nexus between observable and latent variables. The latent variables, estimated through the linear arrangement of observable factors, and the resulting factor are represented by ξj, Xjh, and Yj, respectively. Thus, equation (6) including the estimated and normalized latent variable (ξj) becomes:

(6) $$Y_{j}={\left(\sum_{h=1}^{p_{j}}W_{jh}X_{jh}\right)}^{*}={\left(X_{j}W_{j}\right)}^{*}$$

where Wj*, denotes the weight vector and normalization process. Conversely, it also utilizes the inner estimation techniques, for estimating the correlation between the latent variables. This technique is used to scrutinize the latent variables ξj as well as other connected latent factors and denoted by Zj:

(7) $$Z_{j}={\left(\sum_{i,\beta_{ij}}e_{ij}Y_{i}\right)}^{*}$$

From equation (7) we can identify the coefficients as βij, while the “inner weight” is denoted by e_ij_, measured via the following equation (8):

(8) $$e_{ji}=sign\left(r\left(Y_{j},Y_{i}\right)\right)=\left\{ \begin{array}{c} 1,\left(r\left(Y_{j},Y_{i}\right)>0\right)\\ 0,\left(r\left(Y_{j},Y_{i}\right)=0\right)\\ -1,\left(r\left(Y_{j},Y_{i}\right)<0\right) \end{array}\right.$$

The "sign" is the representation of the “sign function”, while r(Yj, Yi) denotes the concerned coefficient of the outer weight measurement for Yj and Yi. The specification representing the Model 1 is shown below:

(9) $$W_{j}=\frac{1}{n}X_{j}^{T}Z_{j}$$

Specifically equation (9), Wj, Xj, and Zj denote the weight vector, related variable, and variance, respectively. Next, the specification highlighting the model 2 is represented by the following:

(10) $$W_{j}={\left(X_{j}^{T}Z_{j}\right)}^{-1}X_{j}^{T}Z_{j}$$

In equation (10), Wj denotes the coefficients that are estimated via the least square analysis for Zj. To estimate the weights, model 1 and model 2 are used correspondingly, using reflective and formative measurements.

### 3.4 Vector autoregression

Following the norms, the study also checks the main results' robustness by employing an additional technique known as vector autoregression (VAR). It is a valuable and reliable technique when we need to estimate the dynamic linkage between various time series factors [47]. This technique estimates the relationship by regressing the current year values of the variables on their previous year values. The basic assumption behind this technique is that the current values of a variable are always influenced by the previous year's values [48]. As a result, the short-run dynamics and feedback loops are accessible with the help of this technique.

## 4 Data

The primary aim of this study is to assess the factors influencing green investment in China, focusing on the roles of ICT, digital financial inclusion, environmental pressures, and free trade. To accomplish this goal, we compiled time-series data spanning from 1996 to 2022. In Table 1, we provide a comprehensive list of variable abbreviations and their corresponding definitions, along with the sources from which we obtained our data. Following Li et al. [7], our dependent variable in this model is a green investment that is measured using environmental-related technologies (ET). The data on environmental-related technologies is sourced from the OECD. Turning to our independent variables, we first consider ICT. Building on the work of Asongu & Odhiambo [49], we utilize three proxy measures to assess this variable: internet usage as a percentage of the population, mobile cellular subscriptions per 100 people, and fixed telephone subscriptions per 100 people. Our data for internet usage, mobile cellular, and telephone subscriptions comes from the WDI. Next, we examine digital financial inclusion (DFI). Consistent with Ozturk & Ullah [50], we employ two proxy measures: the number of ATMs per 100,000 adults and the percentage of the population holding debit cards. We obtained data for these DFI proxies from GFDD. The third independent variable we consider is free trade (FT), which we gauge through the ASEAN-China free trade agreement. Data for this variable is sourced from the WTO. Following Chen et al. [51], we also measure environmental pollution (EP) using four proxy variables: carbon dioxide (CO2) emissions in kilotons, methane (CH4) emissions in kilotons of CO2 equivalent, nitrous oxide (NO2) emissions in thousand metric tons of CO2 equivalent, and sulfur hexafluoride (SF6) gas emissions, also in thousand metric tons of CO2 equivalent. In addition to these core variables, we include two control parameters in our model: institutional quality (IQ) and gross domestic product (GDP). We gauge institutional quality (IQ) through two measures, political stability (PS) and regulatory quality (RQ), both obtained from the WGI. GDP per capita data, adjusted to constant 2015 US dollars, is also collected from the WDI.

**Table 1:** Variables and abbreviations.

Variables	Description	Abbreviation	Sources
Green investment (GI)	Environmental related technologies (patents)	ET	OECD
Information and Communication Technology (ICT)	Individuals using the Internet (% of population)	Internet	WDI
	Mobile cellular subscriptions (per 100 people)	Mobile	WDI
	Fixed telephone subscriptions (per 100 people)	Telephone	WDI
Digital financial inclusion (DFI)	ATMs per 100,000 adults	ATM	GFDD
	Debit card (% age 15+)	Debit	GFDD
Free trade (FT)	ASEAN-China free trade (dummy)	Ftasean	World Trade Organization
Environmental pollution (EP)	CO2 emissions (kt)	CO2	WDI
	Methane emissions (kt of CO2 equivalent)	CH4	WDI
	Nitrous oxide emissions (thousand metric tons of CO2 equivalent)	NO2	WDI
	SF6 gas emissions (thousand metric tons of CO2 equivalent)	SF6	WDI
Institutional quality (IQ)	Political stability and absence of violence/terrorism: estimate	PS	WGI
	Regulatory quality: estimate	RQ	WGI
Gross domestic product (GDP)	GDP per capita (constant 2015 US$)	GDP	WDI

## 5 Empirical results and discussion

### 5.1 PLS-SEM results

We used PLS-SEM to specify the study mechanism for the current inquiry as it has been effectively applied to manage both simple and difficult frameworks. This also holds true for data that don't fit the analysis's requirements for normality and complexity [52]. While PLS-SEM and the covariance-based technique CBS-SEM are equivalent, PLS-SEM is more precise in identifying and evaluating variable validity. The current study evaluated the measurement model and the structural model using PLS-SEM. The results of the research suggest that estimation of the measurement model may be performed using convergent and discriminant validity approaches.

According to Rehman et al. [53], convergent validity describes how well items from several variables reflect the same variable. Convergent validity evaluates if all questions accurately represent the corresponding predictor. The efficiency of the composite reliability (CR) and average variance extracted (AVE) are assessed for convergence. Furthermore, according to Hair et al. [54], the values for factor loadings, AVE, and CR need to be greater than 0.50, 0.50, and 0.60, respectively. Cronbach's alpha must be higher than 0.60 (Nunnally, 1978). Table 2 shows that the CR score is higher than 0.60 for all variables and that the AVE values are greater than 0.50. Cronbach's alpha value is also higher than the recommended cutoff point of 0.60, while the AVE values are higher than the cutoff value 0.50.

**Table 2:** Constructs’ reliability and convergent validity.

	Cronbach's alpha	Composite reliability (rho_a)	Composite reliability (rho_c)	Average variance extracted (AVE)
GI	0.639	1.000	1.000	1.000
ICT	0.924	1.046	0.949	0.862
DFI	0.975	0.977	0.988	0.976
FT	0.725	1.000	1.000	1.000
EP	0.994	0.994	0.996	0.982
IQ	0.612	0.589	0.592	0.597
GDP	0.943	1.000	1.000	1.000

The constructs (variables) in an SEM are evaluated using the Fornell-Larcker criteria for discriminant validity to determine if they are sufficiently distinct from one another. This is crucial to verify that the constructs are not measuring the same fundamental idea since doing so might generate multicollinearity problems and result in inaccurate parameter estimations in the SEM. To examine the correlations across components in a Fornell-Larcker matrix, square each construct's Average Variance Extracted (AVE). A concept is said to have discriminant validity if its square root of the AVE is more significant than its correlation with other constructs, indicating that it differs from the other constructs [55]. Table 3 demonstrates that the present research satisfies the criteria for discriminant validity. Fornell & Larcker [55] hypothesis states that any "diagonal higher values" are larger than alternate comparable data in identical columns and rows.

**Table 3:** Fornell-Larcker criterion for discriminant validity.

	GDP	GI	DFI	EP	FT	ICT	IQ
GDP	1						
GI	0.994	1					
DFI	0.974	0.966	0.988				
EP	0.992	0.978	0.956	0.991			
FT	0.877	0.866	0.826	0.877	1		
ICT	0.854	0.833	0.920	0.852	0.635	0.928	
IQ	−0.497	−0.45	−0.479	−0.557	−0.374	−0.528	0.705

Table 4 highlights the results of the path analysis on the relationship between ICT, digital financial inclusion, free trade, environmental pressure, and green investment. The path coefficients between DFI and GI, EP and GI, and GDP and GI are positively significant, with values of 0.461, 0.916, and 2.248, respectively. However, the path coefficients between ICT and GI, FT and GI, IQ and GI are positive but insignificant. This finding shows that DFI, EP, and GDP are three factors that help increase green investment in China. This result is consistent with Ding et al. [56] research, which emphasized that digital financial inclusion encourages the adoption of digital payment solutions. These platforms facilitate transactions related to green investments, such as buying and selling sustainable products, paying for clean energy services, or contributing to crowdfunding campaigns for eco-friendly projects. Jiang et al. [57] claimed that digital platforms facilitate the trading of carbon credits and participation in environmental markets. These markets reward organizations and projects for reducing greenhouse gas emissions and adopting sustainable practices. Digital financial inclusion makes it easier for entities to participate in these markets, encouraging green investments that mitigate climate change. Moreover, digital financial inclusion provides easy access to information about green investment opportunities. Our finding infers that digital financial inclusion empowers individuals and communities to engage in green finance, which is essential for addressing environmental challenges and promoting green investment. These findings are also supported by Feng et al. [4], who suggest that digital financial inclusion catalyzes green technology by relaxing the financial limitations on small and medium-sized enterprises. It complements the conventional financial sector and fosters the demand of both consumers and producers, leading to promoting green technological innovation. Digital financial inclusion also promotes green development, a primary driver of green investment, by supporting technological development and the advancement of industrial structures [58].

**Table 4:** Path analysis (PLS-SEM).

	Original sample (O)	Sample mean (M)	Standard deviation (STDEV)	T statistics (|O/STDEV|)	P values
ICT - > GI	0.117	0.104	0.125	0.940	0.347
DFI - > GI	0.461*	0.447	0.272	1.692	0.091
FT - > GI	0.007	0.001	0.116	0.057	0.955
EP - > GI	0.916***	0.887	0.268	3.422	0.001
IQ - > GI	0.001	0.006	0.024	0.028	0.977
GDP - > GI	2.248***	2.225	0.391	5.750	0.000

In support of our EP result, Chen & Ma [59] argued that high levels of environmental pollution lead to stricter environmental regulations. These regulations reduce barriers and increase green investment. Liao [60] described that environmental pollution depletes natural resources and degrades ecosystems. Environmental pressures drive R&D efforts to create new, more sustainable technologies and solutions. These innovations lead to new business opportunities and revenue streams. This finding is also backed by Huang & Lei [61], who noted that environmental pressures increased demand for environmentally friendly products by increasing green investment. This finding is supported by Li et al. [14], who noted that a higher GDP leads to increased consumer and business spending. This creates more demand for green products and services, encouraging businesses to invest in sustainable technologies. With a higher GDP, governments and businesses may allocate more resources to research and development. This leads to innovation in green technologies, making them more affordable and accessible, and driving further investments in environmentally friendly solutions. Economic growth leads to increased infrastructure development, including transportation and energy infrastructure. Governments may choose to invest in green infrastructure projects, such as public transit systems, renewable energy facilities, and energy-efficient buildings, as part of their economic development plans. Higher GDP leads to greater access to capital for businesses. Financial institutions may be more willing to provide loans and investment capital for green projects and initiatives, given the potential for a strong return on investment in a growing economy.

Fig. 1 provides the effects of ICT, DFI, FT, EP, and GI. Our results imply that ICT, DFI, FT, EP, GDP, and IQ directly influence green investment in China. The direct effects of ICT, DFI, FT, EP, and GDP on GI are represented by the estimated values of 0.940, 1.692, 0.057, 3.422, 5.750, and 0.028.

**Fig. 1:** Results of PLS-SEM analysis.

### 5.2 VAR results

Table 5 reports the results of the VAR model. Regarding the green investment equation (GI), our results indicate that for China, ICT, DFI, EP, and FT exhibit statistical significance at the first lag. Specifically, the findings reveal a positive correlation between the first lags of ICT, DFI, EP, and FT with GI. This implies that an increase in the initial values of ICT, DFI, EP, and FT will lead to a corresponding increase in the current level of GI. However, when considering the second lag, the results indicate that ICT, DFI, EP, and FT are statistically insignificant for China concerning green investment.

**Table 5:** VAR results.

	GI	ICT	DFI	EP	FT	GDP	IQ
GI(-1)	0.530	−0.017	0.075	0.006	0.305	0.005	0.082
	[1.467]	[-0.320]	[1.180]	[0.420]	[0.959]	[0.627]	[1.140]
GI(-2)	0.086	−0.043	0.063	−0.010	0.216	0.011	0.094
	[0.220]	[-0.757]	[0.926]	[-0.628]	[ 0.621]	[1.385]	[ 1.212]
ICT(-1)	2.171^b^	1.188^a^	−0.025	−0.102^b^	0.514	0.025^c^	−0.313
	[1.994]	[ 7.509]	[-0.131]	[-2.327]	[ 0.531]	[1.831]	[-1.449]
ICT(-2)	0.938	0.374^c^	−0.025	−0.146^a^	−0.624	0.023	−0.056
	[1.060]	[1.906]	[-0.162]	[-4.113]	[-0.791]	[1.254]	[-0.316]
DFI(-1)	1.274^a^	0.049	0.877^a^	−0.154^b^	0.653	0.006	0.334
	[2.656]	[0.173]	[2.581]	[-1.978]	[ 0.389]	[0.150]	[0.869]
DFI(-2)	1.024	0.055	0.035	0.035	−0.470	0.020	0.916^b^
	[1.271]	[0.198]	[0.102]	[ 0.438]	[-0.268]	[ 0.470]	[2.324]
EP(-1)	2.033^c^	1.277	−0.878	0.871^a^	1.007	0.178	−1.090
	[1.683]	[1.453]	[-0.834]	[3.596]	[ 0.569]	[ 1.399]	[-0.909]
EP(-2)	0.584	1.530	2.172	−0.209	0.837	−0.069	−1.659
	[0.077]	[1.403]	[1.644]	[-0.611]	[0.126]	[-0.435]	[-1.589]
FT(-1)	0.384^b^	0.006^b^	−0.015	0.017	0.396	0.004	−0.069
	[1.994]	[1.994]	[-0.216]	[ 1.084]	[1.158]	[ 0.462]	[-0.943]
FT(-2)	0.075	0.008	0.001	−0.025	−0.235	−0.009	−0.087
	[0.211]	[0.158]	[ 0.007]	[-1.507]	[-0.763]	[-1.278]	[-1.263]
GDP(-1)	1.632	1.902^b^	0.523	−0.820	−1.335	0.239	1.450^b^
	[0.652]	[2.016]	[0.229]	[-1.563]	[-1.065]	[ 0.864]	[2.095]
GDP(-2)	0.151	0.714	−2.270	1.435^b^	0.197	0.495^c^	0.872^b^
	[0.410]	[0.366]	[-0.943]	[ 2.634]	[0.640]	[ 1.720]	[2.176]
IQ(-1)	1.296	0.003	0.023	0.051	0.031	0.024	0.268
	[1.114]	[0.076]	[ 0.115]	[ 1.081]	[0.021]	[ 0.964]	[ 1.152]
IQ(-2)	0.132	0.088	0.048	−0.027	0.325	−0.001	0.127
	[0.085]	[0.493]	[ 0.189]	[-0.444]	[ 0.245]	[-0.029]	[0.427]
C	2.937^c^	0.339	11.31	−2.636	3.787^c^	0.315	1.860^c^
	[1.931]	[0.055]	[1.501]	[-1.536]	[1.944]	[0.342]	[1.945]

Note: T-stats in parentheses.

a p < 0.01.

b p < 0.05.

c p < 0.1.

When estimating a VAR model involving a sequence of causal variables, it is essential to conduct an impulse response function (IRF) analysis. Fig. 2 shows that IRFs results reveal insightful dynamics. For instance, when considering the impact of a one standard deviation shock in ICT on GI, it is evident that this shock initially yields an immediate positive effect. However, this effect diminishes starting from the second year, gradually declining until it becomes statistically insignificant after the fourth year. Similarly, when assessing the influence of a one standard deviation shock in ICT on DFI, the results indicate an instantaneous positive response. This effect intensifies during the first three years, and declines between the third and fifth years, reaching a neutral state from the fifth to the sixth year. Afterward, it experiences a resurgence starting from the seventh year but turns negative beyond the ninth year. In contrast, the impact of a one standard deviation shock in ICT on EP remains insignificant throughout the selected observation period. Additionally, when examining the effect of such a shock on FT, it is noteworthy that it initially lacks significance in the first year but becomes increasingly significant from the second to the third year. Subsequently, it maintains a positive trend until the fourth year but gradually diminishes, eventually becoming insignificant. These findings strongly imply that ICT, DFI, and FT have a substantial and rapidly increasing influence on GI in China. This suggests that these determinants effectively enhance green investment in the country.

**Fig. 2:** Impulse-response functions to ICT shocks.

In Fig. 3, when examining the effect of a one standard deviation shock in DFI on GI, we observe an immediate positive effect in the first two years. Nonetheless, this effect gradually diminishes from the second year onwards, reaching zero in the third year and subsequently becoming statistically insignificant. In Fig. 4, when analyzing the impact of a one standard deviation shock in EP on GI, we note that it initially lacks significance in the first two years. However, this effect gradually turns positive from the second year up to the third year, after which it begins to decline. By the fourth year, it reaches zero, followed by another positive phase until the seventh year. After the seventh year, it returns to zero in the ninth year and eventually becomes statistically insignificant by the tenth year. In Fig. 5, as we investigate the impact of a one standard deviation shock in FT on GI, we find an initial positive effect in the first two years. Nevertheless, this effect progressively diminishes starting from the second year, eventually reaching zero in the third year. It subsequently exhibits a brief positive resurgence from year 3 to year 4 but then declines again from year 4 to year 5, returning to zero and ultimately becoming statistically insignificant.

**Fig. 3:** Impulse-response functions to DFI shocks.

**Fig. 4:** Impulse-response functions to EP shocks.

**Fig. 5:** Impulse-response functions to FT shocks.

## 6 Conclusion and implications

This study investigates the impact of ICT, digital financial inclusion, environmental pressure, and free trade on green investment in China over the period 1996 to 2022. In doing so, we have applied PLS-SEM and VAR approaches to examine the relationship between the variables. The obtained outcomes are reported as follows: The association between ICT, digital financial inclusion, free trade, environmental pressure, and green investment has been investigated using the PLS-SEM approach. According to the structural model's results, the path coefficients between digital financial inclusion and green investment, environmental pressure and green investment, and GDP and green investment are positively significant, implying that these three factors are crucial for boosting green investment in China. In addition, our results suggest that ICT, digital financial inclusion, environmental pressures, free trade, and national income cause green investment to rise in China directly.

Following are the policy suggestions based on our findings. First, to foster energy investments, policymakers must focus on designing and expanding the financial framework. For this purpose, the focus should be on granting tax breaks, subsidies, and funds to firms and ventures that concentrate on sustainability. Strict environmental policies should be implemented and standards should be adopted to tackle environmental deterioration. This may provide equal opportunities to invest in green ventures and ensure that polluting firms are penalized for their acts. Second, policymakers need to invest in the ICT infrastructure constantly, particularly in rural and far-flung areas, to guarantee that all regions of China can reap the fruits of digitalization that support green investment. Third, governments and authorities must try to implement the strategies that are vital in enhancing digital financial inclusion, making sure that households and small enterprises have complete access to digital financial services. In order to achieve this, policymakers must encourage collaborations with the fintech firms and regulatory restructurings. Fourth, concerned authorities must try to promote free trade agreements that support environmental preservation and sustainability. By using their negotiation skills policy makers must incorporate the clauses that are helpful in fostering sustainable initiatives, encourage the use of green technologies, and liberalize markets for green exports. Fifth, public and private collaboration in the form of investment funds for green initiatives must be prioritized. Moreover, these funds must be utilized in promoting R&D activities in the context of green initiatives. Further, the partnership between universities, research centers, and commercial enterprises, could prove beneficial in driving innovation in the green sector. Sixth, policymakers should desive the regulations for the promotion of environmentally friendly technology. Moreover, initiate public awareness campaigns to educate companies and the general public with regard to the benefits of sustainable practices and green investment. Seventh, it is also suggested to prioritize cross-border collaborations to promote the transfer of innovations, investment opportunities, and best practices in the green sector. Eight, policymakers should also try to promote organic farming, sustainable agricultural procedures, and less reliance on chemicals and pesticides in the agriculture sector. They must also enhance the use of “precision agricultural technology” and try to create national action plans and certifications for eco-friendly goods and services. This may prove vital in the promotion of green investment in already sanctioned green ventures and consequently boost customer confidence. Lastly, the development of green infrastructure must also be given priority for promoting green investment and sustainable growth.

Ceraintly the study is a valuable addition to the contemporary, yet some issues need to be addressed in the future. For instance, both PLS-SEM and CB-SEM are used in social sciences and both are good approaches with bit different assumptions. Therefore, it would be more useful if future studies make use of both of these estimators in future studies to compare the results of both estimators. Moreover, the study only considers China as its focused country, which may limit the inferences drawn from the analysis. Thus, it is suggested that future studies perform analysis on other countries and regions to have more valuable insights into the above-stated nexus. Lastly, due to the asymmetric nature of these variables, future studies must also estimate the impacts of ICT, digital financial inclusion, environmental pressures, and free trade on green investment within the non-linear framework.

## Data availability statement

Data will be made available on request.

## CRediT authorship contribution statement

**Jianmin Zhu:** Writing – review & editing, Writing – original draft, Software, Methodology. **Wei Yan:** Writing – review & editing, Writing – original draft, Supervision, Software, Formal analysis. **Junliang He:** Writing – review & editing, Writing – original draft, Validation, Software, Methodology. **Muhammad Hafeez:** Writing – original draft, Supervision, Software, Resources, Methodology, Funding acquisition. **Sidra Sohail:** Writing – original draft, Methodology, Formal analysis, Conceptualization.

## Declaration of competing interest

The authors declare that they have no known competing financial interests or personal relationships that could have appeared to influence the work reported in this paper.
